# Sleep Staging Using Noncontact-Measured Vital Signs

**DOI:** 10.1155/2022/2016598

**Published:** 2022-07-08

**Authors:** Zixia Wang, Shuai Zha, Baoxian Yu, Pengbin Chen, Zhiqiang Pang, Han Zhang

**Affiliations:** ^1^Department of Physics and Telecommunication Engineering, South China Normal University, Guangzhou 510006, China; ^2^Department of Electronic and Information Engineering, South China Normal University, Foshan 528000, China; ^3^Guangdong Provincial Engineering Technology Research Center of Cardiovascular Individual Medicine & Big Data, South China Normal University, Guangzhou 510006, China; ^4^Guangzhou SENVIV Technology Co.,Ltd., Guangzhou 510006, China

## Abstract

As a physiological phenomenon, sleep takes up approximately 30% of human life and significantly affects people's quality of life. To assess the quality of night sleep, polysomnography (PSG) has been recognized as the gold standard for sleep staging. The drawbacks of such a clinical device, however, are obvious, since PSG limits the patient's mobility during the night, which is inconvenient for in-home monitoring. In this paper, a noncontact vital signs monitoring system using the piezoelectric sensors is deployed. Using the so-designed noncontact sensing system, heartbeat interval (HI), respiratory interval (RI), and body movements (BM) are separated and recorded, from which a new dimension of vital signs, referred to as the coordination of heartbeat interval and respiratory interval (CHR), is obtained. By extracting both the independent features of HI, RI, and BM and the coordinated features of CHR in different timescales, Wake-REM-NREM sleep staging is performed, and a postprocessing of staging fusion algorithm is proposed to refine the accuracy of classification. A total of 17 all-night recordings of noncontact measurement simultaneous with PSG from 10 healthy subjects were examined, and the leave-one-out cross-validation was adopted to assess the performance of Wake-REM-NREM sleep staging. Taking the gold standard of PSG as reference, numerical results show that the proposed sleep staging achieves an averaged accuracy and Cohen's Kappa index of 82.42% and 0.63, respectively, and performs robust to subjects suffering from sleep-disordered breathing.

## 1. Introduction

Sleep plays an important role in body recovery, memory, and immunity enhancement, which takes almost one-third of human life [1]. Poor sleep quality usually results in physical and mental health problems, such as fatigue, anxiety, and even death [2]. It has been reported that sleep duration is closely related to mortality [3]. Therefore, long-term sleep quality monitoring is of great significance to protect human health.

Sleep staging is an important characteristic to qualify sleep quality. According to the American Academy of Sleep Medicine (AASM), a complete sleep cycle consists of wake, rapid eye movement (REM), and non-REM (NREM) stages, where the last one can be further divided into N1, N2, and N3 stages [4]. REM and NREM alternate in cycles of about 90 min [5]. NREM, especially deep sleep (N3), is more prominent during the first hours of sleep and is essential toward physical recovery [6, 7]. REM link to dreaming, more prominently during the last hours of sleep, acts toward the recovery of people's mental state [8]. Therefore, a fine-grained classification of Wake-REM-NREM stages is crucial for assessing sleep quality.

Polysomnography (PSG) is the gold standard in the clinic for evaluating sleep quality and diagnosing sleep-related diseases. Physiological signal acquisition during sleep is usually conducted in the hospital since the acquisition process of vital signs is cumbersome. To obtain the physiology signals including electroencephalography (EEG), electrooculography (EOG), electromyography (EMG), electrocardiography (ECG), and respiratory rate [9], a large number of sensors are attached to the skin of patients directly [10], which is impractical for long-term monitoring at home.

Many studies have attempted to classify sleep stages automatically under more natural sleep monitoring conditions by using a limited number of sensing channels. In [11], wrist-actigraphy was used to record body movements during sleep and achieved a sleep/wake classification performance of 77.8%. In [12], the authors took infants as experimental subjects and used wrist-actigraphy to achieve a sleep/wake classification. However, this method has limitations when the subject likes to be quiet in wake period. Motivated by the fact that the autonomic nerves (assessed by heartbeat and respiratory rate) changes in different sleep stages, respiratory inductive plethysmography signals have been used in three-stage classification (i.e., REM/NREM/Wake) and achieved the classification performance of 80.38% [13]. In [14], the authors also considered single-lead ECG heartbeat interval detection and yielded the sleep/wake classification performance of 76%. In order to improve the classification performance, cardiorespiratory features including both the features extracted from heartbeat interval and respiratory are extensively studied [15–19]. Specifically, using ECG sensors, features of heart rate variability in time and frequency domain are fused with the time and effort (fluctuation) features of respiratory signal to aid sleep staging, and the performance of REM/NREM/Wake stages classification was improved to almost 80% [16]. In [20, 21], ECG sensors were used to extract features with respect to heart rate, respiratory rate, and body movement. Although the existing single-lead ECG sensor based methods can achieve satisfactory performance of sleep staging, the acquisition of signals requires physical contact with subjects' skin, which is inappropriate to long-term home monitoring.

In order to solve the discomfort between sensors and skin in the process of signal acquisition, many studies have focused on noncontact monitoring technologies [22]. Using piezoelectric sensors, heart rate was obtained based on noncontact-measured ballistocardiogram (BCG) signals, by which three-stage classification of night sleep is performed [23]. In [24], the authors considered PVDF sensors to record night-sleep physiological signals, including BCG, respiratory signal, and body movements, and then employed long short-term memory (LSTM) neural network [25] to perform end-to-end sleep stage classifications. By analogy, in [26, 27], continuous-wave Doppler radar sensing technology was adopted to distinguish Wake/REM/LightSleep/DeepSleep states and achieved an accuracy of 81% and 66.7% in comparison with PSG standard. Taking radar sensing as the vital sign monitoring system, the authors in [28] evaluated the performance of Wake/REM/NREM sleep staging, where the overall accuracy reached up to 88.4%. Although sleep-related vital signs (i.e., heart rate and respiratory rate) and body movements can be measured by using the existing noncontact sensing devices, the effect of coordinated features between heartbeat interval and respiratory interval in different timescales has not been reported yet.

In order to address the above issues, this paper focuses on a noncontact sensing-based sleep staging for Wake/REM/NREM classification using vital signs recorded by piezoelectric sensors. Specially, the contributions of this paper, in comparison with the existing studied, can be summarized as follows.

1. A noncontact vital signs monitoring system using piezoelectric sensors is deployed, by which both the independent features of heartbeat interval (HI), respiratory interval (RI), body movements (BM), and the coordinated features between HI and RI (a.k.a. CHR) are extracted from the noncontact-measured vital signs and employed for Wake/REM/NREM stage classification. In addition, the effects of features in different timescales on sleep staging are also analyzed.
2. A postprocessing with respect to the fusion of the classified stages is developed to further improve the performance of sleep staging. For validations, 17 all-night experiments were examined simultaneously with PSG. Numerical comparisons demonstrate that the proposed sleep staging achieves average accuracy and Kappa index of 82.42% and 0.63, respectively, and performs robust to subjects suffering from sleep-disordered breathing.

## 2. Materials and Methods

### 2.1. System Setup and Vital Signs Acquisition

For noncontact vital signs acquisition, the noninvasive heart rate and respiratory rate sensing device developed by Guangzhou SENVNV Co. was deployed [29], where the sleep-related physiological signals, including BCG, respiratory signal, and artifact motion can be recorded during night sleep in a noncontact manner. After preprocessing, heartbeat interval, respiratory interval, and body movements are separated, and sleep stage-related features are extracted from the above physiological signals and then fed into machine learning classifiers for sleep stage classification. Finally, an empirical rule-based postprocessing is applied to improve the classification performance.  Figure 1 depicts the framework of the noncontact sleep staging system.

The noncontact vital signs monitoring system deployed in this study consists of a piezoelectric sensor, circuit, and processing modules. As shown in Figure 2, the piezoelectric sensor module is placed under the pillow to perceive the vibration induced by heartbeat, respiratory rate, and body movements. The converted voltage signals are then amplified, sampled at 1 kHz in the circuit module. A 12-bit analog-to-digital conversion (ADC) is conducted before transmission of vital signs from circuit to processing module for offline signal processing and sleep stage classification. For reference, we simultaneously collect EEG, ECG, EOG, and EMG from PSG (Medcare) as the gold standard to evaluate the staging performance.

### 2.2. Noncontact Vital Signs Acquisition

This study involved a total of 10 healthy subjects (7 males and 3 females), who are college students, aged from 21 to 25 years old. All subjects are healthy and have a regular night sleep with an average duration of 6 to 9 hours. In addition, subjects with sleep disorder, smoking habits, intake of medicine, or drinks infecting sleep will not be included. As shown in Table 1, a total of 24 night-sleep experiments are carried out, in which the recorded data in 7 night sleep are invalid due to the collapse of the electrodes of PSG.

### 2.3. Preprocessing of Vital Signs

Since the vital signs measured by the noncontact device are mixed with BCG, respiratory signal, body movements, and noise, preprocessing of vital signs is firstly performed to separate different types of signals for heartbeat interval and respiratory interval detection. The procedures are shown as follows.

First, we remove the power frequency noise by using a band-stop filter with lower and upper cutoff frequencies of 49 Hz and 51 Hz, respectively. Then, we identify body movements (BM) from the processed signal. The reason is that, on the one hand, body movements can significantly affect the detection and analysis of vital signs (i.e., BCG and respiratory signals). On the other hand, as will be illustrated later, body movements signal is an important feature for sleep staging. Unlike [30], body movements (BM) are detected in multi-time-scale procedure. The detailed procedures are as follows. If the peak-to-valley difference (PVD) within a 2 s window is 2.2 times greater than any one of the medians of PVD within a multi-time-scale epochs of 30 s, 60 s, 120 s, and 300 s, the state of 2 s window will be considered as body movement; that is, BM=1; otherwise, BM=0.

Next, we extract BCG from the resulting signals of BM=0. Considering that the spectrum of a typical BCG ranges from 3 Hz to 10 Hz [31], we employ a 2nd-order Butterworth bandpass filter ranges 2.5–10 (Hz) to remove the undesired signal interference and then detect heartbeat interval by using a forward and backward approach [29].

For respiratory interval detection, we remove the detected BCG signal from the recorded vital signs and then separate the respiratory waves directly by using discrete wavelet transform and Sym8 wavelet package at 8 scales [32]. Finally, respiratory interval can be obtained by using peak detection [33].

For validation, a typical example of 20-minute comparison between the noncontact-measured HI and RI and that obtained using BIOPAC MP160, which are recognized as the gold standard in related works. As can be observed from Figure 3, although some errors occur in very limited areas due to the interference of body motion, the noncontact-measured HI and RI are almost indistinguishable from those obtained using ECG and belt sensors. The results demonstrate that the measured HI and RI in a noncontact manner can be further used as features for sleep stage classification.

## 3. Feature Extraction

Using the non-contact-measured vital signs (i.e., HI, RI, and BM signals), we propose feature extraction based on the above independent and coupled vital signs for sleep stage classification. Considering that the relevant features depend on the information of HI and RI, we define the heartbeat interval and respiratory interval in different timescales as

(1) $$\begin{array}{c} {\text{HI}}^{\left(t\right)}=\frac{\sum_{n=1}^{N}\alpha_{n}\beta_{n}I\_h_{n}}{\sum_{n=1}^{N}\alpha_{n}\beta_{n}},\;t=1,3,5,7,9,11,13,15, \end{array}$$

(2) $$\begin{array}{c} {\text{RI}}^{\left(t\right)}=\frac{\sum_{n=1}^{N}\alpha_{n}\beta_{n}I\_r_{n}}{\sum_{n=1}^{N}\alpha_{n}\beta_{n}},\;t=1,3,5,7,9,11,13,15, \end{array}$$

where *N* is the number of heartbeat intervals within *t*-second scale, *I*_*h*_*n*_ and *I*_*r*_*n*_ are the duration of *n*_*th*_ every interval. *α*_*n*_ is the proportion of *I*_*h*_*n*_ or *I*_*r*_*n*_ in time *t*-second (∑_*n*=1_^*N*^*α*_*n*_=1). *β*_*n*_=0 denotes *n*_*th*_ interval occurs in body movement episode; otherwise, *β*_*n*_=1. Specially, if the *t*-second signal is filled with body movement, HI^(*t*)^ and RI^(*t*)^ are defined as the invalid value. Intuitively, the longer the timescale employed for HI and RI detection in (1) and (2), the higher the accuracy of HI and RI, since the relative errors are reduced in the statistical process. By taking advantage of HI and RI in different timescales, independent features with respect to HI and RI can be characterized accordingly.

### 3.1. Independent Features of HI and RI

Table 2 shows all independent features of HI and RI in different timescales. The motivation of independent features extraction with respect to HI and RI is similar to the existing studies [26] since the rhythm of heartbeat and respiratory interval vary in different sleep stages.

Specifically, features {1, 2} and {10, 11} are the mean and coefficient variation of independent HI and RI in different timescales in a 60 s epoch. Features {3–7} and {12–16} further describe the trend of fluctuation with respect to heartbeat interval and respiratory interval over a 60 s epoch by evaluating the ratio of difference in terms of heartbeat interval and respiratory interval percentiles. Motivated by [18, 26], features {8, 9} and {17, 18} are the mean absolute deviation (MAD) and the averaged cumulative difference (ACD) of HI and RI, respectively, which can also reflect the variations of heartbeat interval and respiratory interval in each 60 s epoch.

### 3.2. Coordinated Features between HI and RI

Motivated by the cardiopulmonary coupling technology [34], we propose to characterize the coordinated features between HI and RI, referred to as CHR features, aiming to compensate for the limitations of independent features of HI and RI. Specifically, we define the ratio of HI features over RI features to evaluate the similarities and differences of the coordinated features in different sleep stages. Similar to the independent features class, CHR features also include the ratio of the mean (feature 19), coefficient variation (feature 20), different percentiles (feature 21–31), MAD (feature 32), and ACD of HI and RI (feature 33), as shown in Table 3.

### 3.3. BM Features

As reported by [35], body movement usually occurs in wake and light sleep (a.k.a., N1N2) stages due to sleep posture changes every 5–10 minutes, while rarely appearing in deep sleep (i.e., N3) and REM stages. Motivated by the above facts, we extracted the BM features for sleep stage classification, as shown in Table 4.

Using the above extracted features from the non-contact-measured vital signs, different classifiers including Random Forest (RF) [36], Support Vector Machine (SVM) [37], Decision Tree (DT) [38], *K*-Nearest Neighbor (KNN) [39], and AdaBoost [40] are employed for sleep stage classification.

## 4. Stage Fusion

Since the epoch-by-epoch classification is in a timescale of 60 s, the classified sleep stages are sparse in time domain. According to the AASM, a rule-based postprocessing is proposed to improve the prediction performance by reasonably fusing the sparsely classified epoch-by-epoch sleep stage in time.

(1) Following the rules of AASM, the sequence of sleep stage is from Wake to NREM and then to REM. Based on this fact, the discrete REM labels directly followed by Wake labels are modified to Wake labels.
(2) If the label of a single epoch is different from that of both the previous and the following epochs, it will be relabeled as that of the previous epoch.
(3) For sparsely predicted Wake labels interleaved with either REM or NREM labels, when the proportion of all Wake labeled periods exceeds 80% of a 5-minute timescale, such a 5-minute timescale is fused as Wake stage.
(4) Define *P*_REM_ as the proportion of REM stages over total sleep time; for two adjacent REM labels intervals with other stage labels, we adopt the following fusion criteria:
  - When *P*_REM_ < 5%, two adjacent REM stages less than 20 minutes are fused as one REM stage.
  - When *P*_REM_ > 10%, two adjacent REM stages less than 7 minutes are fused as one REM stage.
  - When *P*_REM_ ∈ [5%, 10%], two adjacent REM stages less than 15 minutes are fused as one REM stage.

## 5. Experimental Results

For the evaluation of sleep staging performance, we adopt leave-one-out cross-validation. To elaborate a little further, classifiers are trained and tested by 16 and 1 samples, respectively, which is repeated until every single sample is tested. The 17 samples based on PSG sleep staging slices form a total of 14666 epochs, where Wake, REM, and NREM stages are 2668, 2562, and 9434 epochs, accounting for 18.19%, 17.47%, and 64.34%, respectively. In this study, we adopt different weights assigned in [24] to avoid overfitting. Similar to [41], we quantify the performance in terms of accuracy and Cohen's Kappa coefficient, respectively, which are given by

(3) $$\begin{array}{c} p_{0}\left(\text{accuracy}\right)=\sum_{\text{class}\left\{\text{Wake},\text{NREM},\text{REM}\right\}}\frac{{\text{TP}}_{\text{class}}}{T},\\ \text{Kappa}=\frac{p_{0}-p_{e}}{1-p_{e}}, \end{array}$$

where *T* and TP_class_ denote the total number of epochs and those correctly classified into the corresponding class and *p*_*e*_ is the hypothetical probability of chance agreement.

(4) $$\begin{array}{c} p_{e}=\sum_{\text{class}\left\{\text{Wake},\text{NREM},\text{REM}\right\}}\frac{{\text{TP}}_{\text{class}}+{\text{FP}}_{\text{class}}}{T}\times \frac{{\text{TP}}_{\text{class}}+{\text{FN}}_{\text{class}}}{T}. \end{array}$$

### 5.1. Effect of Independent and Coordinated Features on Sleep Staging

In order to examine the effectiveness of the extracted features using independent features of HI, RI, BM, and coordinated features between HI and RI, we first evaluate the feature importance using RF classifier [42].  Figure 4 shows the contributions of both the independent features (HI, RI, and BM) and the coordinated features (CHR) to sleep stage classification. As shown in Figure 4, the feature importance of HI class features, RI class features, CHR class features, and BM class features account for 25.4%, 23.2%, 32.6%, 18.8%, respectively. Among them, ACD extracted by HI is the most important feature, revealing that the cumulative difference during sleep is particularly important for sleep staging. It is also noted that CHR features contribute most to sleep stage classification, which demonstrates that coordination between HI and RI is essential to discriminate sleep stages. Specially, Ratio of ACD to CHR performs better, which is consistent with the excellent performance of ACD in the independent features.

Then, we analyze the effect of time resolution with respect to features extraction on sleep staging. As shown in Figure 5, both the accuracy and Kappa tend to increase when *t* < 10 s and then decrease as the timescale increases. A possible explanation to this behavior is that non-contact-measured HI and RI suffers from inevitable errors due to artifact motion and noise, as shown in Figure 3. In this case, increasing the timescale yields a higher accuracy of HI and RI. Benefiting from the increase of timescale when *t* < 10 s, the improvement of feature accuracy improved sleep staging performance. As the timescale grows larger (i.e., *t* > 10 s), it simultaneously reduces the sensitivity with respect to the variation of HI and RI in different timescales, thus leading to a reduced performance. Furthermore, it can be seen that the classification results using CHR features perform better than those without CHR features, demonstrating the effectiveness of the CHR features. The highest accuracy and Kappa are 82.42% and 0.63 when the timescale is 9 s.

### 5.2. Sleep Stage Fusion

Next, we investigate the effect of stage fusion as the postprocessing of classification on sleep staging.  Figure 6 shows the classification performance with and without the proposed sleep stage fusion. It can be seen that the applied stage fusion significantly improves the results, especially in Wake and REM. The accuracy of Wake is increased by 31.6%, and that of REM is increased by 39.9%. The result is reasonable since the epoch-by-epoch classified sleep stages over a specific interval are mapped to an identical sleep stage. Moreover, the accuracy of NREM still maintains a high level of 89.8%, although it may be reduced by 3.2% from 93.0% due to the slight fusion errors in the fusion of Wake and REM.

To further demonstrate the performance improvement of stage fusion, Figure 7 provides a typical example with and without the proposed sleep stage fusion. As can be seen from Figure 7, the proposed stage fusion significantly improves the results.

### 5.3. Wake-REM-NREM Discrimination

We further verify the confusion matrix based on RF classifier, and the result is shown in Figure 8. It can be seen from Figure 8 that the prediction accuracy rates of Wake, REM, and NREM are 67.3%, 53.7%, and 83.7%, respectively. Among them, the dominant error comes from the misclassification between REM and NREM stages. Taking the experimental results into account, the main reason of low accuracy of recognition in REM could be summarized to three aspects. (1) Frequent body movements occur in both Wake and REM stages, leading to a lower accuracy of feature extraction in terms of HI, RI, and CHR, thereby reducing the accuracy of classification. (2) The proportion of REM epochs is lower than that of NREM and Wake. Therefore, the proportion of misclassified epochs of REM in REM is higher than that in the whole sleep stage, whereas the accuracy of the whole system will be less affected.

### 5.4. Validation on Subjects Suffering from Sleep-Disorderd Breathing

As a proof-of-concept with respect to the so-designed sleep staging model, we further consider 7 subjects with sleep-disordered breathing (most of these subjects suffer from mild sleep apnea syndrome), aiming to verify the effectiveness of the proposed design. The data used in the experiment was jointly recorded by The First Affiliate Hospital of Guangzhou Medical University and Guangzhou SENVNV Co., and the experiment has obtained the consent of the subjects, and personal private information is kept confidential. The information of the recruited subjects is listed in Table 5.

Using the proposed scheme with noncontact-measured vital signs, the performance of sleep staging in comparison with PSG is shown in Table 6. It can be seen that the averaged accuracy and Kappa coefficient with respect to the recruited subjects suffering from sleep-disordered breathing are 75.07% and 0.54, respectively. This demonstrates the robustness of the so-designed features and model.  Figure 9 provides a typical sleep stage classification from a subject with sleep-disordered breathing.

## 6. Conclusion

This paper studied feature-aided sleep stage classification using noncontact-measured vital signs. In addition to the analysis of independent features such as HI, RI, and BM, which are characterized from BCG, respiratory rate, and body movements signals in different timescales, we validated through experiments that the coordinated features between HI and RI play an important role in sleep staging. In order to improve the performance of classification, we developed a rule-based postprocessing to fuse the classified results of discrete time dimensions. The experimental results in comparison with PSG demonstrate the effectiveness of the proposed design.

## Figures and Tables

**Figure 1:** The overall architecture of the noncontact sleep monitoring system.

**Figure 2:** The overview of the vital signs monitoring system. (a) The subject simultaneously monitored by both PSG and the noncontact vital signs system. (b) The device of the vital signs monitoring system.

**Figure 3:** An example of comparison between detected HI and RI in a noncontact manner and that obtained by using the gold standard device.

**Figure 4:** Feature importance of HI, RI, BM, and CHR.

**Figure 5:** Accuracy and Kappa in different timescales.

**Figure 6:** The classification performance with and without the proposed sleep stage fusion.

**Figure 7:** (a) Reference sleep stages provided by PSG. (b) Classified sleep stages estimated without stage fusion. (c) Classified sleep stages estimated with stage fusion.

**Figure 8:** Confusion matrix of Wake-REM-NREM sleep stage classification.

**Figure 9:** (a) Reference sleep stages provided by PSG. (b) Classified sleep stages estimated without stage fusion. (c) Classified sleep stages estimated with stage fusion.

**Table 1:** Information of the datasets.

Subject ID	Gender	Age	Weight (kg)	Height (m)	Total (night)	Valid (night)
N1	M	23	65.23	1.70	5	4
N2	M	22	66.52	1.72	4	3
N3	F	21	48.36	1.60	1	0
N4	M	23	70.44	1.74	4	4
N5	F	24	52.62	1.64	1	0
N6	M	23	69.87	1.73	2	2
N7	M	22	62.15	1.67	3	2
N8	F	25	68.53	1.76	1	0
N9	M	22	60.76	1.66	1	1
N10	M	23	67.39	1.75	2	1

**Table 2:** Independent features of HI^(*t*)^(RI^(*t*)^).

Feature index	Feature name	Feature description
1 (10)	Mean	Mean value of HI^(*t*)^(RI^(*t*)^)
2 (11)	CV	Coefficient variation of HI^(*t*)^(RI^(*t*)^): Standard deviation divided by mean
3–7 (12–16)	Inter ratio percentiles	Ratio of percentile A and percentile B of HI^(*t*)^(RI^(*t*)^): (*A*, *B*) ∈ [(100,0), (90,10), (80,20), (70,30), (60,40)]
8 (17)	MAD	Median absolute deviation of HI^(*t*)^(RI^(*t*)^)
9 (18)	ACD	Averaged cumulative difference: the moving average of the absolute difference between the former 30 seconds and the latter 30 seconds of HI^(*t*)^(RI^(*t*)^) for the range from *k* − *q* to *k*+*q* minutes (*q*=2)

**Table 3:** Coordinated features of HI^(*t*)^ and RI^(*t*)^.

Feature index	Feature name	Feature description

19	Ratio of mean	Ratio of mean of HI^(*t*)^ to mean of RI^(*t*)^
20	Ratio of CV	Ratio of CV of HI^(*t*)^ to CV of RI^(*t*)^
21–31	Intra ratio percentiles	Ratio of percentile A of HI^(*t*)^ to percentile B of RI^(*t*)^: (*A*, *B*) ∈ [(100,0), (90,10), (80,20), (70,30), (60,40), (50,50), (40,60), (30,70), (20,80), (10,90), (0,100)]
32	Ratio of MAD	Ratio of MAD of HI^(*t*)^ to MAD of RI^(*t*)^
33	Ratio of ACD	Ratio of ACD of HI^(*t*)^ to ACD of RI^(*t*)^

**Table 4:** Features of BM.

Feature index	Feature name	Feature description
34	Motion ratio	The proportion of body movement in the current epoch
35	Motion nums	The number of periods of successive one-value signal in the current epoch
36	Largest motion ratio	Longest one period in epoch divided by 60
37	Average motion ratio	Motion ratiodivided byMotion nums
38–39	Motion ratio of the previous *n* epochs	The proportion of body movement of epoch located, respectively, *n* ([1, 2]) epochs before the current one
40–41	Motion ratio of the next *n* epochs	The proportion of body movement of epoch located, respectively, *n* ([1, 2]) epochs after the current one

**Table 5:** Information of the subjects with sleep-disordered breathing.

Subject ID	Gender	Age	AHI (times/hour)	Severity	Total (night)	Valid (night)
A1	M	49	10.6	Mild	1	1
A2	F	70	6.3	Mild	2	1
A3	M	70	7.7	Mild	1	1
A4	F	69	8.1	Mild	1	1
A5	M	73	5.9	Mild	2	1
A6	M	50	6.7	Mild	1	1
A7	M	51	7.5	Mild	1	1

**Table 6:** Performance of the sleep-disordered breathing subjects.

Subject ID	Accuracy (%)	Kappa
1	76.07	0.58
2	75.30	0.48
3	65.11	0.39
4	78.49	0.63
5	68.11	0.41
6	79.81	0.67
7	82.62	0.62
Average	75.07	0.54
Std	5.85	0.11

## Data Availability

No datasets are generated during the current study. The datasets analyzed during this work are publicly available.
